# Expression of Cysteine-Rich Secreted Acidic Protein in Multiple Myeloma and Its Effect on the Biological Behavior of Cancer Cells

This article has been retracted.

**DOI:** 10.1155/2021/6101060

**Published:** 2021-10-26

**Authors:** Qiqun Pan, Tangfei Li, Zhangqin Luo, Pengji Pan

**Affiliations:** ^1^Department of Hematology, Zhuji Affiliated Hospital of Shaoxing University, Zhuji, Zhejiang 311800, China; ^2^Department of Hematology, Yongchuan Hospital of Chongqing Medical University, Chongqing 402160, China

## Abstract

The multiple myeloma is a malignant clonal tumor of bone marrow plasma cells that is incurable and inevitably recurrent. The mechanisms of progression include tumor cell metastasis, immune escape, resistance to apoptosis, and malignant proliferation. The cysteine-rich secreted acidic protein is closely related to the growth, development, remodeling, and repair of cells and tissues. In our study, we divided myeloma patients and patients with other blood diseases into groups and measured the cysteine-rich secreted acidic protein (SPARC) content in the serum of different groups of patients as well as the prognostic differences. The U266 cells were transfected with interfering vectors and overexpressed SPARC vectors to determine the physiological functions of MM cells. Our results showed that SPARC was highly expressed in MM and the survival rate of the high SPARC expression group was lower than that of the low expression group. Interfering SPARC vectors inhibited cancer cell proliferation, migration, and invasion and promoted apoptosis. Overexpression of SPARC vectors promoted cancer cell development. SPARC affected the patient's disease development by regulating the biological behavior of the MM cells.

## 1. Introduction

The multiple myeloma (MM) is a malignant clonal tumor of bone marrow plasma cells. Its incidence is second only to lymphoma and is the second most common malignant tumor in hematology [1]. The survival prognosis of MM patients has improved significantly in recent years with the increasing level of treatment, but MM is still incurable and disease recurrence is an inevitable trend in the disease, especially for patients with high biological risk. The main mechanisms of its disease progression include tumor cell metastasis, immune escape, apoptosis resistance, and malignant proliferation of cells that do not depend on the bone marrow microenvironment [2–4]. Therefore, it is still necessary to develop new treatment strategies to solve this dilemma in clinical practice.

At this stage, the main treatment methods for the MM include symptomatic support therapy, high-dose chemotherapy, bone marrow hematopoietic stem cell transplantation, and cellular immunotherapy [5, 6]. In the past decade or so, the selective protease inhibitors (such as bortezomib and carfilzomib) and immunomodulatory drugs (such as lenalidomide) have been widely used, although the median survival period of patients can be extended to six years, but at the same time, the high cost has also increased the financial burden of patients and even caused some patients to refuse treatment [7]. As research on anticancer treatment continues to progress, the exploration of the pathogenesis of the MM has gradually become a focus. Thus, the in-depth study of the molecular mechanism of the MM disease development and the search for molecular targets related to the disease are of great clinical significance for the diagnosis and survival prognosis of patients.

The secreted protein acidic and rich in cysteine (SPARC) is a secreted protein whose physiological function is related to tissue cell growth and development and tissue cell remodeling and repair [8, 9]. Recent studies had shown that SPARC was involved in tumor occurrence, invasion, metastasis, angiogenesis, and inflammation [10]. The SPARC can participate in affecting the growth of a variety of tumor cells by regulating cell cycle, apoptosis, and survival pathways. At the same time, the related proteins involved in regulation in the SPRAC also play a very important role in the antitumor mechanism of drugs, such as Bax, Bcl-2, and PI3K/AKT [11, 12]. In addition, the SPARC expression is increased in many tumors, such as glioma, breast, digestive, and urinary system tumors. The SPARC expression is also related to tumor differentiation, clinical stage, and lymph node metastasis. Clinical studies had shown that the SPARC might be used as a predictor of poor prognosis in gastric cancer. However, there were reports that it had nothing to do with prognosis [13, 14].

The relevant clinical significance of the SPARC expression levels in MM is less reported at present. In this study, we measured SPARC expression levels in MM patients' serum and analyzed the relationship between its expression and clinicopathological characteristics and prognosis; we acquired MM cells to investigate the effect of SPARC expression on the biological behavior of cancer cells and initially explored its clinical significance and related molecular mechanisms.

## 2. Materials and Methods

### 2.1. Clinical Patients Included

The clinical data of 77 MM patients diagnosed and treated in two hospitals from March 2018 to June 2019 were selected as the case group. Inclusion criteria were as follows: (1) the diagnosis of the MM was in accordance with the 2003 International Myeloma Working Group (IMWG) MM diagnostic criteria [15]; (2) the clinical pathology and follow-up data were complete; (3) patients and their families gave informed consent to this study and signed the consent form. Exclusion criteria were as follows: (1) combined history of malignant neoplasm or treatment history, (2) combination of other hematologic diseases such as leukemia and lymphoma, (3) combination of infectious diseases such as pneumonia and *tuberculosis*, (4) neuropsychiatric disorder and inability to cooperate with treatment or follow-up, and (5) receiving other treatments in the past. There were 43 males and 34 females; the age ranged from 36 to 74 years, with an average of (57.9 ± 6.5) years. According to the International Staging System (ISS) [16], there were 13 cases in stage I (*β*2-MG≤3.5 mg/L; albumin>35 g/L), 30 cases in stage II (3.5 mg/*L*<*β*2-MG<5.5 mg/L), and 34 cases in stage III (*β*2-MG≥5.5 mg/L). According to D-S staging, there were 12 cases in stage I, 17 cases in stage II, and 48 cases in stage III. According to diagnostic typing, there were IgG type in 32 cases, IgA type in 25 cases, and light chain type and other types in 20 cases; hemoglobin <100 g/L in 50 cases and hemoglobin ≥100 g/L in 27 cases; blood calcium less than 2.98 mmol/L in 61 cases and not less than 2.98 mmol/L in 16 cases; lactate dehydrogenase less than 245 U/L in 58 cases and not less than 245 U/L in 19 cases. The sixty-three patients with other blood disorders treated at the same time in our hospital were used as the case control group, including 35 males and 28 females; age ranged from 42 to 71 years, with a mean of (55.4 ± 6.1) years. There were 20 cases of non-Hodgkin's lymphoma, 21 cases of acute lymphoblastic leukemia, and 22 cases of chronic myeloid leukemia. The diagnoses were in line with the 2007 “Blood Disease Diagnosis and Efficacy Standards.” Sixty-seven healthy people undergoing physical examinations in our hospital during the same period served as the healthy control group, including 36 males and 31 females, aged 37–72 years, with a mean of (56.8 ± 6.5) years. The differences were not statistically significant (all *P* > 0.05) when comparing the three groups in terms of gender and age and were comparable. This study was approved by the medical ethics committee of our hospital.

### 2.2. Collection and Follow-Up of Clinical Samples

About 5 mL of fasting venous blood was taken from each group in the early morning, anticoagulated with EDTA, and then centrifuged at 4°C and 1200 r/min for 10 min, and finally the serum of the upper layer was stored at −80°C for measurement. The clinical data were collected from the patients. Follow-up began from the date of patient discharge and ended in June 2021. Follow-up was performed as an outpatient or by telephone, once/month, and the follow-up consisted of patient survival, with the follow-up ending at the time of the patient's death event or the end of the follow-up period.

### 2.3. Cell Source and Culture

The MM cell U266 was purchased and placed in Wuhan Pu Nuo Sai Life Technology Co., Ltd., and cultured in RPMI 1640 medium containing 1% double antibody and 10% FBS; the culture conditions were as follows: 37°C and 5% CO_2_. The cell status was observed daily, and the cells were passaged once around 2 d. Cells of logarithmic growth phase were selected for subsequent experiments. Since the U266 cells are suspension cells, centrifugation is an option, and direct passaging is also available.

### 2.4. Cell Transfection and Grouping

The U266 cells were inoculated in 6-well plates at 2.5 × 10^5^/well. 10 *μ*l of SPARC siRNA, SPARC, or control siRNA, oeRNA was diluted in 240 *μ*L of serum-free and antibiotic-free culture medium and gently mixed evenly. 5 *μ*L Lip02000 was diluted in 245 *μ*L serum-free and antibiotic-free culture medium and gently mixed. After 5 minutes, different RNAs were mixed with 5 *μ*L Lip02000 and gently mixed and incubated at room temperature for 20 minutes. The medium was aspirated from the culture plate and the cells were washed twice with serum-free culture medium. In each culture well of the U266 cells, 1500 *μ*L of serum-free culture medium was added. The different complexes (total volume 500 pL) were then added to the culture wells, and the plates were shaken back and forth to distribute them evenly. The cells were incubated in the incubator for 4-6 h, and then the serum-containing culture medium was replaced. The cells were divided into 5 groups: control group, si-NC group, si-SPARC group, oe-NC group, and oe-SPARC group. The control group were control cells without transfection.

### 2.5. qRT-PCR

The U266 cells were inoculated at 2.5 × 10^5^/well in a 6-well plate. The culture medium was aspirated from the plates the next day, and the cells were washed twice with PBS and discarded. Total RNA within cells and patient serum was extracted using the RNAiso method, and RT reactions were performed according to the reverse transcription kit instructions. Based on the obtained cDNA as a template, the primers are as follows: SPARC forward primer (5′-GTGGGCAAAGGGAAGTAACA-3′), SPARC reverse primer (5′-GGGAGGGTGAAGAAAAGGAG-3); GAPDH forward primer (5′-TGCACCACCAACTGCTTAG-3′), and GAPDH reverse primer (5′-GGATGCAGGGATGTTC-3′). The reaction conditions were 95°C for 5 min, 95°C for 30 sec, 56°C for 45 s, 72°C for 45 s, 33 cycles, and 72°C for 10 min. SPARC and GAPDH expression were detected simultaneously in Tanon GIS 2020 imaging analysis photographic system, and GAPDH expression was used as an internal reference. The results were analyzed using the 2^−ΔΔCt^ [17] value method for data analysis, where ΔCt = Ct_SPARC_-Ct_GAPDH_.

### 2.6. CCK-8

The CCK-8 kit was used for the determination of proliferative activity of multiple myeloma cell lines. The logarithmically grown U266 cells were taken and the cell density was adjusted to 10^5^/ml. 100 *μ*l per well was added to a 96-well plate with 5 replicate wells in each group. Then 10 *μ*l of CCK-8 solution was added to each well and the 96-well plate was incubated for 3 h in a dark incubator. The absorbance of each well at 450 nm was measured using an enzyme marker at 24 h, 48 h, and 72 h, respectively. The calculation formula was as follows: inhibition rate = (control group − experimental group)/(control wells − blank wells) × 100%.

### 2.7. Transwell

The U266 cells were taken after 12.5 g/L trypsin digestion and resuspended with serum-free DMEM medium, and the cell density was adjusted to 1 × 10^6^ mL. 200 *μ*L of cell suspension was inoculated in the upper chamber of Transwell, and 800 *μ*L of DMEM medium containing 20% FBS was added to the lower chamber and incubated for 24 h. The chambers were removed, rinsed twice with PBS, then wiped off with cotton swabs to remove the unperforated cells, fixed by 4% paraformaldehyde for 30 min, then stained with crystal violet for 10 min, and observed under a light microscope and the number of migrating cells was counted. When detecting cell invasion, the Transwell upper chambers were precoated with matrix gel before proceeding with the migration assay as described above. The number of membrane penetrating cells was observed and counted under a light microscope.

### 2.8. Flow Cytometry

The apoptosis was detected by flow cytometry Annexin V/PI double-staining assay for comparison of apoptosis rates. The logarithmically grown U266 cells were inoculated in a sterile 6-well plate containing 5 × 10^5^ cells per well in a total volume of 2 ml. The cell suspension was washed twice with PBS and collected. The cells were resuspended with 400 *μ*l PBS, 5 *μ*l AnnexinV and 5 *μ*l PI were added and incubated for 10–15 min at room temperature and protected from light, and the apoptosis rate was detected by cell flow meter. Apoptosis rate = early apoptotic cells + late apoptotic cells.

### 2.9. Statistical Methods

The SPSS 20.0 statistical software was used to analyze the obtained data. The measurement data were expressed as mean ± standard deviation. The *t*-test was used for comparison between groups. Count data were expressed as number of cases or percentages. The *χ*^2^ test was used for comparison between groups. The rank sum test was used for rank data. Kaplan-Meier survival analysis studied the difference in survival prognosis of patients with different SPARC expression in the case group. *P* less than 0.05 indicated that the difference was statistically significant.

## 3. Result

### 3.1. Expression of SPARC in MM Patients

The relative expression of SPARC in serum of healthy control group, case control group, and MM group was (1.00 ± 0.11), (1.04 ± 0.13), and (3.11 ± 0.21), respectively. The relative expression of SPARC in serum of MM group was significantly higher than that of case control group and healthy control group (*P* < 0.05), but there was no significant difference between case group and healthy group, as shown in Figure 1.

### 3.2. The Relationship between SPARC Expression and Clinicopathology of MM Patients

The relative expression of SPARC in serum of patients with different ISS stages and hemoglobin levels in MM group was significantly different (*P* < 0.05). The main manifestation was that the relative expression of SPARC was high in patients with ISS stage III and hemoglobin <100 g/L. There was no significant difference in the relative expression of SPARC in serum of patients with different age, sex, D-S stage, diagnosis type, serum lactate dehydrogenase, and serum calcium level (*P* > 0.05), as shown in Table 1.

### 3.3. The Relationship between SPARC Expression and Prognosis of MM Patients

In this study, 77 patients in the MM group were followed up for three years, during which 2 cases were lost to follow-up. By the end of the follow-up period, 23 patients had died. Based on the mean SPARC expression of serum 3.11, 39 cases were classified as the high SPARC expression group and 36 cases were classified as the low SPARC expression group. The 3-year overall survival rates of the high SPARC expression group and the low SPARC expression group were 56.41% (22/39) and 83.33% (30/36), respectively. Kaplan–Meier survival analysis results indicated that the 3-year survival rate of SPARC low expression group was significantly higher than that of SPARC high expression group (log-rank = 4.452, *P*=0.035), as shown in Figure 2.

### 3.4. The Effect of SPARC on MM Cell Viability

To detect the influence of SPARC on the biological behavior of MM cells, we transfected MM cells and detected SPARC expression by qRT-PCR. Compared with the control group, SPARC expression in the si-NC group and oe-NC group had no obvious change (*P* > 0.05), while SPARC expression in the si-SPARC group decreased significantly, while SPARC expression in the oe-SPARC group significantly increased, with statistical significance (*P* < 0.05). The result was shown in Figure 3(a), indicating successful transfection of MM cells. The MM cell viability detection by CCK-8 showed that the cell viability of the si-SPARC group was lower than that of the si-NC group, and the cell viability of the oe-SPARC group was higher than that of the oe-NC group. The differences were statistically significant (*P* < 0.05), as shown in Figure 3(b).

### 3.5. The Effect of SPARC on MM Cell Migration and Invasion

The results of Transwell showed that the migration and invasion ability of MM cells in the si-SPARC group was weaker than that in the si-NC group, while that in the oe-SPARC group was stronger than that in the oe-NC group, and the differences were statistically significant (*P* < 0.05), as shown in Figures 4(a) and 4(b).

### 3.6. The Effect of SPARC on MM Cell Apoptosis

The apoptosis rate of MM cells detected by flow cytometry showed that the apoptosis rate of the si-SPARC group was higher than that of the si-NC group, while that of the oe-SPARC group was lower than that of the oe-NC group, and the difference was statistically significant (*P* < 0.05), as shown in Figure 5.

## 4. Discussion

MM is a kind of hematological malignancy with malignant clonal proliferation of plasma cells in bone marrow. Every year, 63,000 people worldwide die from this disease. MM has long incubation period, is difficult to diagnose, and has different clinical manifestations, which seriously affects the quality of life of patients [18]. At present, the treatment of MM includes chemotherapy, immunoregulatory factors, proteasome inhibitors, and autologous hematopoietic stem cell transplantation. Although the survival time of patients is prolonged, they cannot be cured completely. It has been reported that the complete remission rate of MM patients treated with conventional VAD or MP combined chemotherapy is less than 10% [19]. Molecular biology studies have found that the pathogenesis of MM is a gradual change process. Therefore, finding new molecular therapeutic targets and exploring the molecular mechanism related to MM may be a direction to discover new therapeutic strategies and improve the prognosis of MM.

SPARC protein is a highly conserved extracellular matrix protein, whose main functions are to destroy cell adhesion, regulate cell differentiation, prevent cell spreading, inhibit cell response to some growth factors, regulate the production of extracellular matrix and matrix metalloproteinases, and influence neovascularization [8]. Recent studies have shown that SPARC is related to the clinical data of tumor patients [20]. In order to explore the expression of SPARC in MM patients and its relationship with clinical features, we detected the serum of 77 MM patients and analyzed their clinical data. It was found that SPARC was highly expressed in the serum of MM patients and correlated with different ISS stages and hemoglobin levels. We speculated that SPARC can affect the clinical features of patients, which may be related to increased cell vitality and more invasiveness. The relationship between SPARC and tumor prognosis is still controversial. Some studies suggest that the increase of SPARC expression is related to the decrease of survival rate [21], and some studies suggest that the upregulation of SPARC can improve the prognosis of tumor patients [22]. In our study, we found that the 3-year survival rate of MM patients with low serum SPARC expression was significantly higher than that of patients with high serum SPARC expression. It is concluded that the high expression of SPARC is related to the poor prognosis of MM patients. However, due to the limited sample size and time included in this study, there may be meaningful results with the increase of sample size and the extension of follow-up time.

The biological behavior of cancer cells plays an important role in the occurrence and development of MM, affecting the metastasis, recurrence, and even prognosis of patients. Excessive proliferation of MM cells leads to bone lesions, renal function damage, anemia, hypercalcemia, and other clinical manifestations, which seriously threatens human health. SPARC plays an important role in biological regulation during the occurrence and development of diseases and can affect the biological processes such as differentiation and development, proliferation, apoptosis, and metastasis of cancer cells [9]. Therefore, we speculate that SPARC may also play an important regulatory role in the progression of MM disease. To verify this conjecture, we purchased the MM cell line U266 and explored its influence on cell viability, migration, invasion, and apoptosis by interfering and overexpressing SPARC expression in U266 cells. CCK-8, Transwell, and flow cytometry were used to detect the biological behavior of MM cells. It was found that, compared with the si-NC group, the vitality, migration, and invasion ability of cells in the si-SPARC group decreased, while the apoptosis rate increased. The cell viability, migration, and invasion ability of the oe-SPARC group were increased compared with those of the oe-NC group, but the apoptosis rate decreased. These results suggested that SPARC may be involved in regulating the biological behavior of MM cells and may affect the development of patients' diseases by regulating the biological behavior of MM cells.

To sum up, SPARC is highly expressed in MM, which is related to the clinical characteristics and prognosis of patients. Interference or overexpression of SPARC vector can affect the biological behaviors of MM cells, such as proliferation, migration, invasion, and apoptosis.

## Figures and Tables

**Figure 1:** The expression of SPARC in MM patients. *Note.* Compared with healthy control group, ^*∗*^*P* < 0.05; compared with case control group, ^#^*P* < 0.05.

**Figure 2:** The relationship between the expression of SPARC and the prognosis of MM patients.

**Figure 3:** The effect of SPARC on the viability of MM cells. *Note.* Compared with the control group, ^*∗*^*P* < 0.05; compared with the si-NC group, ^#^*P* < 0.05; compared with the oe-NC group, ^+^*P* < 0.05.

**Figure 4:** The effect of SPARC on the migration and invasion of MM cells (200×). *Note.* Compared with the si-NC group, ^#^*P* < 0.05; compared with the oe-NC group, ^+^*P* < 0.05.

**Figure 5:** The effect of SPARC on MM cell apoptosis. *Note.* Compared with the si-NC group, ^#^*P* < 0.05; compared with the oe-NC group, ^+^*P* < 0.05.

**Table 1:** The relationship between the expression of SPARC and the clinicopathology of MM patients.

Items	*N*	SPARC	*t*/*F* value	*P* value
Age (years)				
≤60	35	3.05 ± 0.18	1.828	0.072
>60	42	3.13 ± 0.20		

Gender				
Male	43	3.08 ± 0.21	1.194	0.236
Female	34	3.02 ± 0.23		

D-S staging				
Phase I	12	3.06 ± 0.18	0.836	0.438
Phase II	17	3.14 ± 0.23		
Phase III	48	3.07 ± 0.20		

ISS staging				
Phase I	13	3.04 ± 0.16	4.371	0.016
Phase II	30	3.17 ± 0.19		
Phase III	34	3.25 ± 0.26		

Diagnostic typing				
IgG type	32	3.08 ± 0.20	0.264	0.769
IgA type	25	3.07 ± 0.19		
Light chain type and others	20	3.11 ± 0.17		

Lactate dehydrogenase (U/L)				
<245	58	3.10 ± 0.19	0.194	0.847
≥245	19	3.09 ± 0.21		

Blood calcium (mmol/L)				
<2.98	61	3.11 ± 0.20		
≥2.98	16	3.12 ± 0.17		

Hemoglobin (g/L)				
<100	50	3.30 ± 0.25	2.966	0.004
≥100	27	3.13 ± 0.22		

## Data Availability

The data used and analyzed during the current study are available from the corresponding author on reasonable request.
